# Rhotekin 2 silencing inhibits proliferation and induces apoptosis in human osteosarcoma cells

**DOI:** 10.1042/BSR20181384

**Published:** 2018-11-21

**Authors:** Xiong Wang, Lei Zhang, Wenji Wang, Yuchen Wang, Ye Chen, Ruimin Xie, Xiang Li, Yongping Wang

**Affiliations:** 1 Department of Orthopedics, The First Hospital of Lanzhou University, Lanzhou 730000, China; 2 Guangdong Provincial Key Laboratory of Malignant Tumor Epigenetics and Gene Regulation, Sun Yat-sen Memorial Hospital, Sun Yat-sen University, Guangzhou, China; 3 Department of Orthopedics, Guangzhou Huaxin Orthopedic Hospital, Guangzhou, China; 4 Division of Rheumatology, Penn State Hershey College of Medicine, Hershey, PA, U.S.A.; 5 First Clinical Medical College, Lanzhou University, Lanzhou, China

**Keywords:** apoptosis, cell cycle, osteosarcoma, proliferation, RTKN2

## Abstract

Human osteosarcoma is the most frequent primary malignant of bone, and often occurs in adolescents. However, molecular mechanism of this disease remains unclear. In the present study, we found that the level of Rhotekin 2 (RTKN2) was up-regulated in osteosarcoma tissues and cell lines. In addition, silencing of RTKN2 of human osteosarcoma cell lines U2OS, inhibited proliferation, and induced G_1_ phase cell cycle arrest via reducing the level of the cyclin-dependent kinase 2 (CDK2). Furthermore, RTKN2 knockdown in the U2OS cells induced apoptosis by increasing the level of Bax and decreasing the level of Bcl2. These results suggested that RTKN2 is involved in the progression of human osteosarcoma, and may be a potential therapeutic target.

## Introduction

Human osteosarcoma often occurs in adolescents, and is frequent primary malignant of bone [1–3]. Although the development of novel multimodal therapeutics during last decades, the prognosis with osteosarcoma is generally poor [4,5]. Therefore, it is critical to understand the molecular mechanisms of human osteosarcoma to identify a novel effective therapeutic target.

The Rho GTPases are members of the RAS superfamily, regulating many cellular processes including cell differentiation, survival, gene transcription, and cell-cycle progression [6]. Rhotekin (RTKN), a Rho effector, was initially isolated as a scaffold protein interacting with GTP-bound form of Rho [7]. Two RTKN proteins, RTKN1 and RTKN2, with the same Rho GTPase-binding domain, have homologs in mammals [8]. Previous studies have shown that RTKN2 is overexpressed in bone marrow [9]. In addition, knockdown of RTKN2 in human CD4^+^ T cells reduces viability [10], which associates with apoptosis [11–13]. These findings suggest an involvement of RTKN2 in tumor progression. However, up to now, the biological functions of RTKN2 in human osteosarcoma remain to be unclear.

The present study investigated the expression of RTKN2 in osteosarcoma tissues and human osteosarcoma cell lines. RTKN2 silencing on cell proliferation of human osteosarcoma cells, and the potential mechanism was examined. The results may offer effective therapeutic target for human osteosarcoma.

## Materials and methods

### Tissue samples and cell culture

Osteosarcoma tissues and matched adjacent tissues were obtained form 15 patients who underwent surgery between 2014 and 2018 at the First Hospital of Lanzhou University. The present study had already gotten approval from the institutional ethics committee of the First Hospital of Lanzhou University.

The human osteosarcoma cell lines, MNNG/HOS and U2OS, used in the present study were purchased from the Cell Bank of Chinese Academy of Sciences (Shanghai, China) and cultured in RPMI-1640 (Gibco, Rockville, MD, U.S.A.) at 37°C in 5% CO_2_-humidified air. Human normal osteoblast cells hFOB 1.19 (American Type Culture Collection, Manassas, VA, U.S.A.) were cultured in Dulbecco’s modified Eagle’s medium (DMEM, Gibco, Rockville, MD, U.S.A.) according to the providing sources. All culture media were supplemented with 10% FBS, 100 mg/ml penicillin G, and 50 μg/ml streptomycin (Invitrogen; Thermo Fisher Scientific, Inc., Waltham, MA, U.S.A.).

### RNAi

SiRNAs (Sangon Biotech Co., Ltd., Shanghai, China) were used against RTKN2 that target different regions of its mRNA (siRTKN2-1, 5′-GCU UUG GUA GUA CCC AUU ATT-3′; siRTKN2-2, 5′-GCU UUG GUA GUA CCC AUU ATT-3′; siRTKN2-3, 5′-CCU UCU GGC AGC AUU UCU UTT-3′). The cells were transfected with siRNA (50 nM) using Lipofectamine 3000 (Invitrogen; Thermo Fisher Scientific, Inc., Waltham, MA, U.S.A.), according to the protocol. Nonspecific siRNA was used as a negative control (si-control, 5′-UUC UCC GAA CGU GUC ACG UTT-3′), and silencing of RTKN2 was confirmed by real-time PCR and western blot assay. After 48 h of transfection, cells were collected for further analysis.

### Cell Counting Kit-8 assay

Cell proliferation assay was performed by Cell Counting Kit-8 (CCK-8; Beyotime Institute of Biotechnology, Haimen, Jiangsu, China). Briefly, the cells were seeded in 96-well culture plates at an initial density of 5 × 10^3^ cells per well. At specified time points (at 0, 1, 2, 3, 4, 5, and 6 days), 10 μl of CCK-8 was added to each well, then incubated for 2 h at 37°C. Absorbance was detected in a microplate reader (ELx800; Bio-Tek Instruments, Inc., Winooski, VT, U.S.A.) at 450 nm. Each group had five replicated wells.

### Colony formation assay

The cells were dissociated into single-cell suspension, and re-inoculated in the six-well plates at a cell density of × 10^2^ cells/well, 48 h after siRNA transfection. The cells were incubated for 2 weeks until the clone spots were visible. Then the cells were washed and fixed with 4% paraformaldehyde for 10 min and washed three times with PBS solution. Then the cells were stained with Crystal Violet for 15 min, followed by washing with PBS, and then photographed under light microscope (Olympus, Japan) after dried at room temperature. The number of colonies (>50 cells/colony) was counted. At least three independent experiments were performed.

### Flow cytometry for cell cycle analysis

Cell cycle assay was measured by flow cytometry (Beckman Coulter, Brea, CA, U.S.A.). Briefly, approximately 1 × 10^6^ cells were collected and washed twice with PBS, then fixed in 70% cold ethanol (precooling at −20°C) for 4 h at least, and followed by incubation with RNase (50 mg/ml) for 15 min, and then incubated with propidium iodide (PI; Sigma, St. Louis, MO, U.S.A.) for 30 min at room temperature. The cells were then analyzed by flow cytometry. Four replicates were included for each group in the experiment.

### Apoptosis assay by flow cytometry

Apoptosis assay was performed by using Annexin V FITC Apoptosis Detection kit with PI (Biovision, Inc, Mountain View, CA, U.S.A.) according to the protocol. The cells were collected and resuspended in 400 μl binding buffer, containing 5 μl Annexin-V FITC and PI, following which the cells were incubated for 15 min at room temperature in the dark prior to flow cytometry. Data were analyzed with FlowJo 7.0 software (FlowJo LLC., U.S.A.). Four replicates were included for each group in the experiment.

### Hoechst 33258

Nuclear morphology of apoptotic cells was also examined by Hoechst 33258 (Beyotime Institute of Biotechnology, Haimen, Jiangsu, China). Briefly, the cells were fixed with 4% paraformaldehyde for 30 min and washed three times with PBS. Then cells were stained with 10 mg/l Hoechst 33258 for 10 min at room temperature in the dark place. Morphologic changes in apoptotic nuclei were observed under fluorescence microscope (Olympus, Japan). The cells with condensed chromatin and shrunken nuclei were classified as apoptotic cells. Apoptosis was assessed by counting the number of apoptotic cells in five random fields per slide.

### Real-time PCR

Total RNA was extracted by using RNAiso Plus reagent (Takara Biotechnology Co. Dalian, China) following the protocol. Then cDNAs were synthesized using the Primescript RT Master Mix (Takara Biotechnology Co., Dalian, China). Real-time PCR were undertaken by using the SYBR Premix ExTaq II (Takara Biotechnology Co. Dalian, China). The condition was as follows: 94°C for 30 s, followed by 40 cycles of 95°C for 5 s, and 60°C for 30 s in a 10-μl reaction volume. The primers are described in Table 1. The relative gene expression was calculated according to the 2^−ΔΔ*C*T^ method, with glyceraldehyde-3-phosphate dehydrogenase (GAPDH) as an internal control.

**Table 1:** Primer sequences used in the present study

Gene	Primer sequence
*RTKN2*	Forward: 5′-ACAGTTCGCGTTGGAGATGGAG-3′
	Reverse: 5′-GTCGAGCATTGCACACCATGAG-3′
*Bax*	Forward: 5′-ATCCAAGACCAGGGTGGTT-3′
	Reverse: 5′-ATCTGGAAGAAGATGGGCTG-3′
*Bcl-2*	Forward: 5′-GGCCTCTGTTTGATTTCTCC-3′
	Reverse: 5′-AGTGAAGTCAACATGCCTGC-3′
*CDK2*	Forward: 5′-CTCCTGGGCTCGAAATATTATTCCACAG-3′
	Reverse: 5′-CCGGAAGAGCTGGTCAATCTCAGA-3′
*GAPDH*	Forward: 5′-CACCCACTCCTCCACCTTTG-3′
	Forward: 5′-CCACCACCCTGTTGCTGTAG-3′

### Western blot assay

Western blot analyses were performed according to standard procedures [14]. The total proteins were obtained by using RIPA lysis buffer (Beyotime Institute of Biotechnology, Haimen, Jiangsu, China). After centrifugation at 14000 rpm for 30 min at 4°C, the supernatant was collected and the concentration was measured by the BCA assay (Beyotime Institute of Biotechnology, Haimen, Jiangsu, China). Total protein (50 μg) was separated using SDS-PAGE (Beyotime Institute of Biotechnology, Haimen, Jiangsu, China), then transferred to PVDF membrane, which was blocked with 5% skim milk for 1 h and then incubated with primary antibodies against RTKN2 (1:1000; Abcam, Cambridge, MA, U.S.A.), Bax (1:1000; Abcam, Cambridge, MA, U.S.A.), and Bcl2 (1:1000; Abcam, Cambridge, MA, U.S.A.) at 4°C overnight. GAPDH (1:5000; Cell Signaling Technology, Danvers, MA, U.S.A.) was used as a loading control. The membranes were subsequently washed three times with TBS with Tween 20 (TBST), and then incubated with horseradish peroxidase–conjugated secondary antibody (1:10000) for 1 h at room temperature. The bands were visualized with ECL imaging (Beyotime Institute of Biotechnology, Haimen, Jiangsu, China) and imaged using a VersaDoc Imaging System (Bio-Rad Laboratories Co., Ltd. Hercules, CA, U.S.A.). The integral optical density (IOD) value of each band was performed.

### Statistical analysis

Statistical analysis was performed by SPSS 16.0 (IBM, Armonk, NY, U.S.A.) software. We used GraphPad Prism 7.0 (version X; La Jolla, CA, U.S.A.) for image editing. Data are expressed as the mean ± S.D. of at least three independently performed experiments. The significant differences between groups were analyzed using Student’s *t*test. A *P*-value of <0.05 was considered to indicate a statistical significance.

## Results

### RTKN2 is overexpressed in human osteosarcoma

To determine the role of RTKN2 in osteosarcoma, we first detected the levels of RTKN2 in osteosarcoma tissues and matched adjacent tissues by real-time PCR and western blot, which suggested that the mRNA and protein expression levels were higher in osteosarcoma tissues than in matched adjacent tissues (Figure 1A, B). We next detected the levels of RTKN2 in two human osteosarcoma cell lines and a normal osteoblast cell line by real-time PCR and western blot. Compared with the normal osteoblast cell line, RTKN2 overexpression was detected at both the mRNA and protein levels in osteosarcoma cell lines (Figure 1C, D). The results showed that RTKN2 may play an important role in osteosarcoma. The expression level of RTKN2 was markedly higher in U2OS cells, so we selected U2OS cells to investigate the function of RTKN2 in human osteosarcoma.

**Figure 1:** RTKN2 was overexpressed in human osteosarcoma (**A**) The expression level of RTKN2 was up-regulated in human osteosarcoma tissues by real-time PCR and western blot (**B**). (**C**) The mRNA and (**D**) protein expression levels of RTKN2 were assessed by real-time PCR and western blot in osteosarcoma cell lines (MNNG/HOS and U2OS) and a human normal osteoblast cell line (hFOB 1.19). *P<0.05.

### RTKN2 silencing inhibits proliferation of human osteosarcoma U2OS cells

To explore the functional significance of RTKN2 in human osteosarcoma, RTKN2 siRNAs were used to silence RTKN2 in human osteosarcoma U2OS cells with higher RTKN2 level. The knockdown efficiency of siRNAs for RTKN2 was confirmed through comparison with negative control (si-control) at mRNA and protein levels (Figure 2). Amongst the siRNAs tested, siRNA-3 generated the most consistent knockdown results and was thus chosen for subsequent studies. RTKN2 mRNA (Figure 2A) and protein (Figure 2B, C) expression levels were significantly decreased after transfection with RTKN2 siRNAs in U2OS cells. Next, a CCK-8 assay (Figure 3A) was used to detect cell proliferation. A 6-day growth curve analysis showed that the RTKN2 silencing significantly inhibited the proliferation of human osteosarcoma U2OS cells. A colony formation assay (Figure 3B, C) was carried out to determine the colony forming capacity of osteosarcoma cells after the knockdown of RTKN2. The number of colonies was obviously decreased in the RTKN2-knockdown group than control group.

**Figure 2:** Silencing of RTKN2 by siRNA in human osteosarcoma U2OS cells (**A**) Real-time PCR and (**B and C**) western blot analyses revealed that the expression levels of RTKN2 were significantly inhibited by RTKN2 siRNAs in the U2OS cells. Amongst the three siRNAs tested, siRNA-3 generated the most consistent knockdown results and was thus chosen for subsequent studies. *P<0.05.

**Figure 3:** Knockdown of RTKN2 inhibits proliferation and growth of human osteosarcoma U2OS cells (**A**) Analysis using CCK-8 identified significant inhibition in the proliferation of U2OS cells. (**B and C**) The growth of cells was determined by colony formation assay. *P<0.05.

### RTKN2 silencing induces G_1_ cell cycle arrest in human osteosarcoma U2OS cells

The present study then determined the possible inhibitory effect of RTKN2 knockdown on cell cycle distribution. Cell cycle changes in response to RTKN2 knockdown were analyzed using flow cytometry. In the absence of RTKN2 siRNA, the populations of cells in the G_1_, S, and G_2_ phases were determined. Transfection of the cells with siRNA was accompanied by a concomitant increase in the G_1_ phase population in the U2OS cells, as shown in Figure 4. These results suggested that RTKN2 knockdown induced G_1_ cell cycle arrest in human osteosarcoma U2OS cells, which may be associated with the inhibition of proliferation.

**Figure 4:** Silencing of RTKN2 arrests cell cycle at the G_1_ phase (**A and B**) Flow cytometric analysis identified significant arrest at the G_1_ phase of the cell cycle in the U2OS cells. *P<0.05.

### Knockdown of RTKN2 induces cell apoptosis of human osteosarcoma U2OS cells

Decreased cell proliferation induced by RTKN2 knockdown may be a consequence of increased cell death. Thus, we examine the effects of RTKN2 on cell apoptosis. Annexin V/PI staining was performed. The cells undergoing apoptosis was increased in the RTKN siRNA-treated U2OS cells compared with the control group (Figure 5A, B). These results were further confirmed by a morphological analysis by Hoechst 33258. As shown in Figure 5C, D, nuclei morphological change was observed. The control cells exhibited uniformly dispersed chromatin, normal organelle, and intact cell membrane. However, silencing of RTKN2 induces apoptosis of human osteosarcoma U2OS cells, with featured typical characteristics of apoptosis, including the condensation of chromatin, the shrinkage of nuclei, and the appearance of a few apoptotic bodies. These data suggested that RTKN2 may have an important anti-apoptotic role in human osteosarcoma.

**Figure 5:** Knockdown of RTKN2 induces cell apoptosis (**A and B**) U2OS cells were stained with Annexin-V FITC/PI, and apoptotic cells were analyzed using flow cytometry. (**C**) Morphological changes associated with apoptosis were examined by Hoechst 33258 staining. (**D**) The apoptotic index was determined by (number of positively stained cells/total number of cells) × 100%. White arrowheads in the images indicate the nuclei of apoptotic cells (magnification, ×200). *P<0.05.

### Silencing of RTKN2 inhibits the expression levels of cell cycle-associated and anti-apoptosis protein

RTKN2 knockdown resulted in significant decreases in the levels of cyclin-dependent kinase 2 (CDK2) in the U2OS-siRTKN2 cells than the control group (Figure 6B, C, E). Silencing of RTKN2 inhibited the expression of cell cycle-associated proteins, which may have contributed to the induction of G_1_ cell cycle arrest. In addition, the data indicated the silencing of RTKN2 inhibited the expression of anti-apoptosis protein Bcl2 and increased the expression of pro-apoptosis protein Bax (Figure 6A, C, D), which resulted in cell apoptosis. It is thought that the ratio of the pro-apoptotic protein Bax and the anti-apoptotic protein Bcl-2 plays a crucial role in the control of the intrinsic pathway of apoptosis. We therefore reasoned that the cell death induced by RTKN2 knockdown might be due to changes in this ratio (Figure 6F). These results further demonstrated that RTKN2 had the potential anti-apoptosis in human osteosarcoma cells.

**Figure 6:** The expression of several crucial cell cycle and apoptosis-related proteins in U2OS cells after transfection with RTKN2-siRNA (**A**,**B**) Real-time PCR and Western blot analysis (**C**) showed significant increase in the expression of Bax, and significantly decreased expression of Bcl-2 and CDK2. *P<0.05. (**D**,**E**) The results were quantitatively analyzed by densitometry. (**F**) Ratio of Bax/Bcl-2 protein level. *P<0.05.

## Discussion

In recent years, despite the development of new multimodal therapeutics, the prognosis with human osteosarcoma is generally poor. Therefore, it is important to identify additional potential treatments. RTKN are members of a Rho effector protein [15]. The involvement of RTKN2 in several types of cancer has been reported [16–18]. In this study, we primarily found that RTKN2 was critical for osteosarcoma cell survival. We analyzed the mRNA and protein levels of RTKN2, and found that the level of RTKN2 was up-regulated in osteosarcoma tissues and human osteosarcoma cells. Functional study by knockdown of RTKN2 helped us illustrate the important role of RTKN2 in human osteosarcoma that RTKN2 silencing resulted in suppressed growth of human osteosarcoma cells and impaired colony formation ability of human osteosarcoma cell. In addition, G_1_ phase arrest and apoptosis were induced after RTKN2 knockdown, which could partly explain the reduced cell viability of RTKN2 silencing U2OS cells. These results implied that this protein RTKN2 functions as an oncogene and were necessary for human osteosarcoma cell survival.

The Rho GTPases regulate many cellular processes including cell survival and cell cycle progression [6]. RTKN2, a novel identified Rho–GTPase effector protein, was initially isolated as a scaffold protein interacting with GTP-bound form of Rho [7]. Dysfunction of RTKN2 has been reported to play an important role in numerous types of cancer. Previous studies have shown that RTKN2 is overexpressed in bone marrow [9]. In addition, knockdown of RTKN2 in human CD4^+^ T cells reduces viability [10], which associates with apoptosis [11–13]. Pang et al. [19] showed that the inhibitory effect of RTKN2 silencing on the proliferation of colon cancer cells may be partially realized by inhibiting the Wnt/β-catenin signaling pathway. Several studies have shown that RTKN2 played a critical role in apoptosis, which was dependent on NF-kB signaling and expression of Bcl-2 [9,16,20]. And Lin et al. [21] indicated that miR-181 inhibited the tumorigenesis of ovarian cancer through RTKN2-NF-kB pathway. These findings suggest an involvement of RTKN2 in tumor progression.

Cell cycle components are often abnormal in malignancy, thus resulting in uncontrollable proliferation [22,23]. In this study, RTKN2 silencing induced cell cycle arrest in G_1_ phase in the human osteosarcoma U2OS cells, which indicated that the inhibition of proliferation in human osteosarcoma cells was associated with the cell cycle arrest. The cell cycle distribution is regulated by aberrant CDKs [24]. For example, colon cancer cells proliferate in the absence of CDK2 efficiently, whereas knockdown of CDK2 in osteosarcoma cells prevents their proliferation [25,26]. In our study, the levels of the CDK2 were significantly decreased in the osteosarcoma U2OS-siRTKN2 cells, which was in complete agreement with the results showing the induction of cell cycle arrest in G_1_ phase in the U2OS-siRTKN2 U2OS cells. This indicated the presence of correlation between RTKN2, cell cycle progression, and the regulation of DNA replication in human osteosarcoma cells.

Apoptosis is the process of cell death characterized by cell shrinkage and nuclear condensation. The anti-apoptotic, Bcl-2, is localized in the outer mitochondrial membrane, and the pro-apoptotic factor, Bax, resides in the cytosol. Translocation of Bax to the mitochondrial membrane might lead to an increase in mitochondrial permeability. In addition, it is thought that the ratio of Bax and Bcl-2 plays a crucial role in the control of the intrinsic pathway of apoptosis. In the present study, silencing of RTKN2 increased level of the Bax and the ratio of Bax/Bcl2, and decreased expression of Bcl-2. The flow cytometry data and Hoechst 33258 indicated that the silencing of RTKN2 resulted in notable induction of apoptosis, which was in keeping with previous studies on hepatocellular carcinoma [27], bladder cancer [28], leukemic [29], and colon cancer [19].

In conclusion, our study showed that RTKN2 was overexpressed in human osteosarcoma. Silencing of RTKN2 inhibited proliferation of human osteosarcoma cells, arrested the cell cycle in G_1_ phase, and induced human osteosarcoma cells apoptosis. These data suggested that RTKN2 may provide an effective treatment target in the human osteosarcoma.

## Abbreviations

CCK-8: Cell Counting Kit-8
CDK: cyclin-dependent kinase
GAPDH: glyceraldehyde-3-phosphate dehydrogenase
PI: propidium iodide
RTKN: Rhotekin

## References

[1] PoletajewS., FusL. and WasiutynskiA. (2011) Current concepts on pathogenesis and biology of metastatic osteosarcoma tumors. Ortop. Traumatol. Rehabil. 13, 537–545 10.5604/15093492.971038 22248458

[2] Endo-MunozL., EvdokiouA. and SaundersN.A. (2012) The role of osteoclasts and tumour-associated macrophages in osteosarcoma metastasis. Biochim. Biophys. Acta 1826, 434–442 2284633710.1016/j.bbcan.2012.07.003

[3] TaoZ.W. and ZouP.A. (2018) Adenovirus small interfering RNA targeting ezrin induces apoptosis and inhibits metastasis of human osteosarcoma MG-63 cells. Biosci. Rep., 38, BSR20180351 10.1042/BSR2018035129899165PMC6131204

[4] YaoC., WeiJ.-j., WangZ.-y. (2012) Perifosine induces cell apoptosis in human osteosarcoma cells: new implication for osteosarcoma therapy? Cell Biochem. Biophys. 65, 217–227 10.1007/s12013-012-9423-523015227

[5] AllisonD.C., CarneyS.C., AhlmannE.R. (2012) A meta-analysis of osteosarcoma outcomes in the modern medical era. Sarcoma 2012, 704872 10.1155/2012/704872 22550423PMC3329715

[6] BishopA.L. and HallA. (2000) Rho GTPases and their effector proteins. Biochem. J. 348, 241–255 10.1042/bj3480241 10816416PMC1221060

[7] ReidT., FuruyashikiT., IshizakiT. (1996) Rhotekin, a new putative target for Rho bearing homology to a serine/threonine kinase, PKN, and rhophilin in the rho-binding domain. J. Biol. Chem. 271, 13556–13560 10.1074/jbc.271.23.13556 8662891

[8] CollierF.M., Gregorio-KingC.C., GoughT.J. (2004) Identification and characterization of a lymphocytic Rho-GTPase effector: rhotekin-2. Biochem. Biophys. Res. Commun. 324, 1360–1369 10.1016/j.bbrc.2004.09.205 15504364

[9] CollierF.M., LovingA., BakerA.J. (2009) RTKN2 induces NF-kappaB dependent resistance to intrinsic apoptosis in HEK cells and regulates BCL-2 genes in human CD4(+) lymphocytes. J. Cell Death 2, 9–23 10.4137/JCD.S2891 26124677PMC4474337

[10] Gregorio-KingC.C., GoughT., van der MeerG.J. (2004) Mechanisms of resistance to the cytotoxic effects of oxysterols in human leukemic cells. J. Steroid Biochem. Mol. Biol. 88, 311–320 10.1016/j.jsbmb.2003.12.007 15120425

[11] AupeixK., WeltinD., MejiaJ.E. (1995) Oxysterol-induced apoptosis in human monocytic cell lines. Immunobiology 194, 415–428 10.1016/S0171-2985(11)80108-7 8749234

[12] Ayala-TorresS., MollerP.C., JohnsonB.H. (1997) Characteristics of 25-hydroxycholesterol-induced apoptosis in the human leukemic cell line CEM. Exp. Cell Res. 235, 35–47 10.1006/excr.1997.3630 9281350

[13] Gregorio-KingC.C., CollierF.M., BoltonK.A. (2002) Effect of oxysterols on hematopoietic progenitor cells. Exp. Hematol. 30, 670–678 10.1016/S0301-472X(02)00833-0 12135663

[14] ZhangL., LiY., QiaoL. (2015) Protective effects of hepatic stellate cells against cisplatin-induced apoptosis in human hepatoma G2 cells. Int. J. Oncol. 47, 632–640 10.3892/ijo.2015.3024 26035065

[15] YinT.-Y., HsiaoY.-W., PengW.-H. (2014) Abstract 4435: overexpression of Rhotekin confers gastric cancer cells resistance to interferon-α-mediated growth inhibition. Cancer Res. 72, 4435–4435 10.1158/1538-7445.AM2012-4435

[16] MyouzenK., KochiY., OkadaY. (2012) Functional variants in NFKBIE and RTKN2 involved in activation of the NF-kappaB pathway are associated with rheumatoid arthritis in Japanese. PLoS Genet. 8, e1002949 10.1371/journal.pgen.1002949 23028356PMC3441678

[17] LiW., WuY.F., XuR.H. (2014) miR-1246 releases RTKN2-dependent resistance to UVB-induced apoptosis in HaCaT cells. Mol. Cell. Biochem. 394, 299–306 10.1007/s11010-014-2108-1 24880483

[18] Gregorio-KingC., GoughT., CollierF. (2003) RTKN2 - A novel gene differentially expressed in CD34+cells from umbilical cord blood, normal and AML bone marrow. Exp. Hematol. 31, 206–207

[19] PangX., LiR., ShiD. (2017) Knockdown of Rhotekin 2 expression suppresses proliferation and induces apoptosis in colon cancer cells. Oncol. Lett. 14, 8028–8034 2925018710.3892/ol.2017.7182PMC5727621

[20] LiuC.A., WangM.J., ChiC.W. (2004) Rho/Rhotekin-mediated NF-kappaB activation confers resistance to apoptosis. Oncogene 23, 8731–8742 10.1038/sj.onc.1208106 15480428

[21] LinZ., LiD., ChengW. (2018) MicroRNA-181 functions as an antioncogene and mediates NF-kappaB pathway by targeting RTKN2 in ovarian cancers. Reprod. Sci., 10.1177/193371911880586530309296

[22] WangS., BianC., YangZ. (2009) miR-145 inhibits breast cancer cell growth through RTKN. Int. J. Oncol. 34, 1461–1466 19360360

[23] SevliS., UzumcuA., SolakM. (2010) The function of microRNAs, small but potent molecules, in human prostate cancer. Prostate Cancer Prostatic Dis. 13, 208–217 10.1038/pcan.2010.21 20585343

[24] MalumbresM. and BarbacidM. (2005) Mammalian cyclin-dependent kinases. Trends Biochem. Sci. 30, 630–641 10.1016/j.tibs.2005.09.005 16236519

[25] van den HeuvelS. and HarlowE. (1993) Distinct roles for cyclin-dependent kinases in cell cycle control. Science 262, 2050–2054 10.1126/science.8266103 8266103

[26] TetsuO. and McCormickF. (2003) Proliferation of cancer cells despite CDK2 inhibition. Cancer Cell 3, 233–245 10.1016/S1535-6108(03)00053-9 12676582

[27] WeiW., ChenH. and LiuS. (2016) Knockdown of Rhotekin 2 expression suppresses proliferation and invasion and induces apoptosis in hepatocellular carcinoma cells. Mol. Med. Rep. 13, 4865–4871 10.3892/mmr.2016.5113 27081789

[28] LiaoY.X., ZengJ.M., ZhouJ.J. (2016) Silencing of RTKN2 by siRNA suppresses proliferation, and induces G1 arrest and apoptosis in human bladder cancer cells. Mol. Med. Rep. 13, 4872–4878 10.3892/mmr.2016.5127 27082503

[29] Dat leT., MatsuoT., YoshimaruT. (2012) Identification of genes potentially involved in bone metastasis by genome-wide gene expression profile analysis of non-small cell lung cancer in mice. Int. J. Oncol. 40, 1455–1469 2229404110.3892/ijo.2012.1348

